The article "Effect of Probiotics Therapy on Nonalcoholic Fatty Liver Disease" was published in 2022. Journal: Comput Math Methods Med.

# Effect of Probiotics Therapy on Nonalcoholic Fatty Liver Disease

**DOI:** 10.1155/2022/7888076

**Published:** 2022-05-30

**Authors:** Yuanshe Huang, Xiaodong Wang, Lai Zhang, Ke Zheng, Jie Xiong, Jing Li, Chunlei Cong, Zhaomiao Gong, Jingxin Mao

**Affiliations:** ^1^Anshun University, Guizhou, Anshun 561000, China; ^2^College of Pharmaceutical Sciences, Southwest University, Chongqing 400715, China; ^3^Chongqing Medical and Pharmaceutical College, Chongqing 400030, China; ^4^Department of Endocrine and Breast Surgery, The First Affiliated Hospital of Chongqing Medical University, No. 1 Youyi Road, Yuzhong District, Chongqing 400016, China; ^5^Department of Pharmacy, Ministry of Education Key Laboratory of Child Development and Disorders, National Clinical Research Center for Child Health and Disorders/Chongqing Key Laboratory of Pediatrics/Children's Hospital of Chongqing Medical University, Chongqing 400014, China

## Abstract

**Objective:**

Nonalcoholic fatty liver disease (NAFLD) is the most prevalent chronic liver disease in the world. The pathogenesis of NAFLD is complex and multifactorial. Clinical studies have shown that alterations in the gut microbiota play a key role in NAFLD. The purpose of this study was to analyze the effect of probiotic supplementation on the treatment of NAFLD patients based on various indicators.

**Methods:**

We conducted a meta-analysis investigating the relationship between NAFLD and probiotic supplementation. Embase, PubMed, and Web of Science databases were searched by computer, and then, eligible studies were identified. Finally, a total of high-quality randomized controlled trials were selected involving 1403 participants. Meta-analysis was performed using the RevMan 5.3 software which was systematically searched for works published through Dec. 1, 2021, in the present study.

**Results:**

The meta-analysis results showed that the probiotics supplementation improved hepatocyte injury and significantly reduced the level of ALT (*P* = 0.00001), AST (*P* = 0.0009), GGT (*P* = 0.04), TG (*P* = 0.01), LDL-C (*P* = 0.0005), HDL-C (*P* = 0.0002), insulin (*P* = 0.003), IR (*P* = 0.03), BMI (*P* = 0.03), TNF-*α* (*P* = 0.03), and CRP (*P* = 0.02), respectively, in NAFLD patients.

**Conclusion:**

The present study suggests that probiotics therapy may improve liver enzyme levels, regulated lipid metabolism, reduced insulin resistance, and improved inflammation in NAFLD patients. It supports the potential role of probiotics supplementation in the treatment of NAFLD.

## 1. Introduction

Nonalcoholic fatty liver disease (NAFLD) was always considered to be a disorder caused by excessive deposition of fat in liver cells in addition to alcohol and other definite factors [1]. The incidence of NAFLD is increasing year by year, and it has become the most common cause of chronic liver disease in both developed and developing countries [2]. The NAFLD disease mainly includes nonalcoholic fatty liver (NAFL) and nonalcoholic steatohepatitis (NASH) which commonly associated cirrhosis and liver cancer [3]. It was reported that 2%-3% of NAFLD patients and 15%-20% of NASH patients may finally develop into cirrhosis or even liver cancer [4]. Although the complex pathogenesis of NAFLD has not been fully elucidated, its pathogenesis is mainly related to metabolic abnormalities, such as insulin resistance (IR), type 2 diabetes, visceral obesity, and abnormal metabolism of blood lipids [5]. An international expert consensus statement was issued by a multinational expert group to change the name of NAFLD to a new definition of metabolic fatty liver disease (MAFLD) in 2020 [6]. The “two-hit theory” was the first hypothesis proposed for the pathogenesis of NAFLD. The “first hit” is characterized by lipid accumulation in the liver due to IR [7] while the “second hit” is characterized by lipid peroxidation, secretion of proinflammatory cytokines, and mitochondrial dysfunction that determines disease progression [8, 9]. It is currently known that these mechanisms are not sufficient to explain all NAFLD pathogenesis, so the “multiple parallel hit theory” has received increasing attention. According to this concept, several processes including adipose tissue-derived signaling, gut barrier dysfunction, genetic factors, endoplasmic reticulum stress, and related signaling networks may work together to contribute to the progression of steatosis to NASH development [10].

The article "Effect of Probiotics Therapy on Nonalcoholic Fatty Liver Disease" was published in 2022. Journal: Comput Math Methods Med.

It was reported that the human gut microbiota has emerged as a major participant in human health and disease. The gut and liver “communicate extensively” through the biliary tract, portal vein, and systemic circulation. This bidirectional connection is called the “gut-liver axis.” The liver becomes a key first-line immune organ [11]. Previous studies have shown that the intestinal flora may play a regulatory role in NAFLD and other metabolic diseases through the “gut-liver axis” [12], and it has also been found in clinical practice that patients with NAFLD may easily suffered from imbalance of gut microbiota and microbial metabolic dysfunction. The metabolic function of microorganisms in the tract is disordered, and the number of pathogenic bacteria significantly increases [13]. The liver receives a variety of gut-derived signals that including bacterial products, environmental toxins, and food antigens and normally strikes a balance between immunity and tolerance that is critical to its function. Even in the absence of pathogens, changes in the gut microbiota brought about disruption of intestinal homeostasis which leading to disturbances in immune status and various liver diseases. Excessive immune responses may also cause sterile liver inflammation, chronic inflammation, and liver disease-related cancer [14]. Nowadays, there is a lack of effective drugs for the treatment of NAFLD both domestically and abroad. The main treatment is to improve lifestyle and metabolic disorder. Among the commonly used clinical drugs, the therapeutic effect of vitamin E on IR is not clear, and it will increase the risk of stroke. Pioglitazone may significantly increase the patient's weight, and obecholate will lead to abnormal lipid metabolism [15].

The article "Effect of Probiotics Therapy on Nonalcoholic Fatty Liver Disease" was published in 2022. Journal: Comput Math Methods Med.

Probiotics are known as nonpathogenic living microorganisms which may affect the health of the host by regulating the intestinal microbiota, producing antibacterial substances, improving epithelial barrier function, and reducing intestinal inflammation [16]. At birth, the gastrointestinal tract is sterile. Within a few months after birth, a relatively stable microbial population was established. This kind of rich, diverse, and dynamic intestinal flora usually has a complex symbiotic relationship with mucosal eukaryotic cells. Intestinal microbial imbalance is closely related to the occurrence and progress of NAFLD. It was reported that probiotics may improve the risk factors of NAFLD by affecting the intestinal microbiota [17]. With the in-depth study of probiotics, many clinical and basic trials have been proved that probiotics are a potential treatment for NAFLD. In the present study, we conducted a meta-analysis of the clinical literature of probiotics in the treatment of NAFLD in recent 10 years, so as to provide evidence-based medical basis for the clinical treatment of NAFLD.

## 2. Methods

### 2.1. Search Strategy

Systematic review and meta-analysis were conducted according to Preferred Reporting Items for Systematic Reviews and Meta-Analyse (PRISMA) guidelines to ensure the reliability and integrity of data and conclusions [18]. A comprehensive literature search was conducted on the database (Embase, PubMed, and Web of Science) using the keyword words as follows: “non alcoholic fatty liver disease” OR “NAFLD” OR “nonalcoholic fatty liver disease” OR “nonalcoholic fatty liver” OR “nonalcoholic steatohepatitis” OR “NASH” OR “NAFL” AND “Lactobacillus” OR “probiotics” OR “synbiotic”. The publication time range of the literature is from January 1, 2011, to December 1, 2021.

### 2.2. Selection Criteria

We followed the methods of Mao et al. in 2020 and 2022, respectively [19, 20]. The following selection criteria had been used for the decision-making process.

The article "Effect of Probiotics Therapy on Nonalcoholic Fatty Liver Disease" was published in 2022. Journal: Comput Math Methods Med.

Inclusion criteria are as follows: (1) the clinical trials in the literature were randomized controlled trials (RCTs); (2) the participants were patients with NAFLD who were not restricted by age, sex, or race; (3) the intervention was probiotics; (4) studies that directly assess the effects of probiotics based on any outcome measure; and (5) complete outcome data were available to assess treatment effects.

Exclusion criteria are as follows: (1) the trial was not a RCT trial; (2) patients with hepatic steatosis or fibrosis due to other causes, such as viral hepatitis, autoimmune hepatitis, drug-induced hepatitis, and liver disease due to genetic causes, were all excluded; (3) the experimental measures were interfered with by other therapeutic measures; (4) literature was conference case reports, letters to the editor, editorials, or abstract; (5) studying period beyond 10 years; and (6) insufficient data or only from big data.

### 2.3. Data Extraction

The data of the included literature were extracted using the preset table by two researchers (Table 1), including the first author, the year of publication, case number, intervention time, diagnostic method, probiotic ingredients, control group, and Newcastle Ottawa Scale (NOS).

### 2.4. Literature Quality Evaluation

Three researchers independently evaluated the quality of the included literature according to Cochrane Collaboration tool (version 5.1.0), including whether the research object was generated by random method, whether the distribution scheme was hidden, whether blind method was used, data integrity, whether there was selective report, and other bias.

### 2.5. Heterogeneity, Sensitivity Test, and Publication Bias Analysis

The *Q* test was used to analyze the heterogeneity of the pooled effect sizes, and the results were expressed by *I*^2^ using the RevMan 5.3 software. If there is homogeneity among studies (*P* > 0.05 or *I*^2^ ≤ 50%), the fixed-effect model is used for analysis; otherwise, if there is heterogeneity (*P* ≤ 0.05 or *I*^2^ > 50%), subgroup analysis should be performed to reduce heterogeneity as much as possible. If the cause of heterogeneity is not found, the random effect model is used for meta-analysis. Sensitivity analysis was carried out by comparing the difference between point estimation and interval estimation of combined effect values in different effect models. Begg's test was used for publication bias analysis; it indicates that there is no obvious publication bias if *P* > 0.1.

### 2.6. Statistical Evaluation

Meta-analysis was performed using the RevMan 5.3 software. When the measurement methods or units of the effect of the same intervention were exactly the same, the mean difference (MD) pooled statistic was selected. When different measurement methods or units were used for the effect of the same intervention, the standard mean difference (SMD) was selected as the pooled statistic. All data were analyzed with 95% confidence interval (CI). Data analyses were performed using the *Q* test and *I*^2^ statistic to detect heterogeneity. Using a forest plot to describe the results, with *P* values less than 0.05 considered statistically significant. The NOS was used to assess the quality of the research. In addition, Begg funnel plots have been used to search for viable publication bias.

The article "Effect of Probiotics Therapy on Nonalcoholic Fatty Liver Disease" was published in 2022. Journal: Comput Math Methods Med.

## 3. Results

Through the search strategy, 24 studies that met the criteria in the past 10 years were finally included, including a total of 1403 patients. The flow chart of the study selection process is presented in Figure 1. The study population includes children and adults, with the diagnosis method of ultrasonic examination and liver biopsy combined with clinical biochemical indicators. The probiotics preparations included in the literature mainly include *Lactobacillus*, *Bifidobacterium*, *Enterococcus*, *Streptococcus*, *Bacillus*, and *Lactococcus*. The basic characteristics of the included studies and the quality assessment of the literature are listed in Table 1. The quality of the literature was assessed using the Cochrane Collaboration tool. The evaluation criteria of NOS are based on whether the definition and diagnosis of the disease are appropriate, whether the pathology is representative, whether the selection of control is reasonable, whether there are reliable data sources, whether double-blind analysis is used, etc. A total score of 1 to 4 was considered low quality, and a score of 5 to 9 was considered high quality. A total of 24 articles were all high-quality, and none of the articles had a high risk of bias. The related factors for probiotics therapy on NAFLD patients are presented in Table 2.

### 3.1. Effects of Probiotics on Liver Enzymes in NAFLD Patients

The effect of supplementing probiotics on alanine aminotransferase (ALT) was explored in 19 included literatures in the study. The heterogeneity test results showed that heterogeneity exists in the literature (*I*^2^ = 71% > 87%, *Q*test*P* < 0.00001). Therefore, random effects were used to meta-analysis. The MD value of the 19 literature summary was -7.25; the 95% CI was among -10.11 to -4.39, *Z* = −4.97, and *P* < 0.00001 (Figure 2(a)). The effect of supplementing probiotics on aspartate aminotransferase (AST) was investigated in 18 included literatures. The heterogeneity test results investigated that heterogeneity exists in the present study (*I*^2^ = 71% > 50% and the *Q* test *P* < 0.00001). Qualitative, random effects were selected for meta-analysis. The MD value of the 18 literature summary was -3.53; the 95% CI was among -5.62 to -1.44, *Z* = 2.69, and *P* = 0.0009 < 0.05 (Figure 2(b)). The effect of probiotics on *γ*-glutamyltransferase (GGT) was studied in a total of 9 literatures. The heterogeneity assessment results found that heterogeneity exists in the literature (*I*^2^ = 92% > 50% and the *Q* test *P* = 0.00001). Therefore, random effects were selected for meta-analysis. The MD value of the 9 literatures was -2.27; the 95% CI was among -4.49 to -0.05, *Z* = 2, and *P* = 0.04 < 0.05 (Figure 2(c)). It was suggested that probiotics supplementation in the treatment of NAFLD patients may improve hepatocyte injury and intrahepatic biliary obstruction and significantly reduce the level of ALT, AST and GGT.

The article "Effect of Probiotics Therapy on Nonalcoholic Fatty Liver Disease" was published in 2022. Journal: Comput Math Methods Med.

### 3.2. Effect of Probiotics on Lipid Metabolism in Patients with NAFLD

Effect of probiotics supplement on triglyceride (TG) was studied in 15 literatures. The heterogeneity test results revealed that heterogeneity exists in the inclusive literatures (*I*^2^ = 53% > 50%, *P* = 0.008 < 0.05 in *Q* test). Random effects were selected for meta-analysis. The MD value of 15 literatures was -0.42; the 95% CI is among -0.53 to 0.05, *Z* = 1.59, and *P* = 0.01 (Figure 3(a)). Effect of probiotics supplementation on low density lipoprotein (LDL-C) was investigated in 15 studies. The heterogeneity test results explored that heterogeneity exists in the present study (*I*^2^ = 90% > 50% and *P* < 0.00001 of *Q* test). Random effects were selected for meta-analysis. The MD value of 15 literatures is -1.38; the 95% CI is among -2.15 to -0.60, *Z* = 3.47, and *P* = 0.0005 < 0.05 (Figure 3(b)). Effect of probiotics on high density lipoprotein (HDL-C) was investigated in 18 literatures. The test results of statistical heterogeneity for the meta-analysis of literatures are heterogeneity that exists (*I*^2^ = 53% > 50%and*P* < 0.00001of*Q*test). Random effects were selected for meta-analysis. The MD value of 18 literatures is -19.92; the 95% CI is among -30.56 to -9.29, *Z* = 3.67, and *P* = 0.0002 < 0.05 (Figure 3(c)). It was indicated that probiotics supplementation in the treatment of NAFLD patients may significantly reduce the level of TG, LDL-C, and HDL-C.

### 3.3. Effect of Probiotics on Blood Glucose-Related Indexes in Patients with NAFLD

Effect of probiotics on insulin resistance (IR) was studied in the present study. Test results of statistical heterogeneity for the meta-analysis of literatures (*I*^2^ = 89% > 50%and*P* < 0.00001of*Q*test). Random effects were selected for meta-analysis. The MD value of 13 literatures is -0.61; the 95% CI is -1.02 to -0.21, *Z* = 2.98, and *P* = 0.003 < 0.05 (Figure 4(a)). Effect of probiotics on insulin was explored in 11 literatures. The heterogeneity test results revealed that heterogeneity exists in the present study (*I*^2^ = 86% > 50% and *P* < 0.00001 of *Q* test). Therefore, the random effects were selected for meta-analysis. The MD value of 11 literatures is -1.27; the 95% CI is among -2.39 to -0.15, *Z* = 2.23, and *P* = 0.03 < 0.05 (Figure 4(b)). Effects of probiotics on blood glucose (GLU) were studied in total of 10 articles. The heterogeneity test results showed that no heterogeneity found in the literature (*I*^2^ = 0% < 50% and *P* = 0.45 > 0.1 of *Q* test), and the fixed effects were selected for meta-analysis. The MD value of 10 literatures is -0.03; the 95% CI is among -0.32 to 0.25, *Z* = 0.23, and *P* = 0.82 (Figure 4(c)). The above suggests that probiotics supplementation in the treatment of NAFLD may significantly reduce the levels of insulin and IR.

The article "Effect of Probiotics Therapy on Nonalcoholic Fatty Liver Disease" was published in 2022. Journal: Comput Math Methods Med.

### 3.4. Effects of Probiotics on BMI and Inflammation in NAFLD Patients

The effect of probiotics supplementation on body mass index (BMI) was investigated in 24 literatures. The heterogeneity test results revealed that heterogeneity exists in the present study (*I*^2^ = 89% > 50% and the *Q* test *P* < 0.00001). A random effect was selected for meta-analysis. The MD value of the 24 literature pooled was -0.80; the 95% CI was among -1.51 to -0.08, *Z* = 2.18, and *P* = 0.03 < 0.05, suggesting that probiotics treatment of NALFD may significantly reduce the BMI of patients (Figure 5(a)). Effect of probiotics supplementation on tumor necrosis factor-*α* (TNF-*α*) was explored in 10 included literatures. The test results of statistical heterogeneity for the meta-analysis were *I*^2^ = 99% > 50% and *Q* test *P* < 0.00001, respectively (heterogeneity exists), and random effects were selected for meta-analysis. The MD value of the 10 articles was -2.43; the 95% CI was among -6.56 to 1.71, *Z* = 1.15, and *P* = 0.03 (Figure 5(b)). Effect of probiotics supplementation on C-reactive protein (CRP) was investigated in 6 included literatures. The heterogeneity test results revealed that no heterogeneity exists in the studied researches (*I*^2^ = 0% < 50% and *Q* test *P* = 0.15 > 0.1). Therefore, fixed effects can be selected for meta-analysis. The MD value of the six literature pools was -1.06; the 95% CI was among -1.94 to -0.18, *Z* = 2.36, and *P* = 0.02 < 0.05 (Figure 5(c)). It was suggested that supplementing probiotics in the treatment of NALFD may significantly decreased the levels of BMI, TNF-*α*, and CRP.

The article "Effect of Probiotics Therapy on Nonalcoholic Fatty Liver Disease" was published in 2022. Journal: Comput Math Methods Med.

### 3.5. Results of Heterogeneity, Sensitivity Test, and Bias Publication Analysis

Due to the obvious heterogeneity of some indicators, further subgroup analysis showed that there was no correlation between the country of publication and the heterogeneity, while the intervention time of the study group was related to the heterogeneity of the literature. Sensitivity analyses were performed by comparing the differential changes in point estimates and interval estimates of pooled effect sizes when different effect models were compared. The results showed that there was no change in the conclusions of each indicator, indicating that the results of the meta-analysis of each indicator in this study were stable. Cochrane funnel plot was used to explore the publication bias. There is no obvious asymmetric distribution exhibits in Figure 6 which indicating that there was no publication bias.

## 4. Discussion

NAFLD usually refers to the excessive accumulation of triglycerides in hepatocytes ≥ 5% without heavy drinking (less than 20 or 30 g/day for women and men, respectively) or other liver diseases such as viral, autoimmune, metabolic, or drug-induced [21]. NAFLD pathology is mainly characterized by the deposition of fat particles in the liver, ballooning of hepatocytes, increase of inflammatory cells, and infiltration of liver tissue. It is the manifestation of systemic metabolic syndrome in liver tissue. Although NAFLD is a benign disease, it may lead to liver fibrosis, liver cirrhosis, and even liver cancer [22]. NAFLD is becoming an important public health problem because it is now the main cause of chronic liver disease worldwide. About 80 million to 100 million adults suffer from NAFLD in the United States alone. Approximately 20% of NAFLD patients in the United States have nonalcoholic steatohepatitis (NASH) [23]. In addition, the prevalence of NAFLD is about 15% in adults while 1.3% of children and adolescents in China. The incidence rate of NAFLD in 2 nonalcoholic health volunteers in Shanghai was 6.1% for 2 years [24].

There are 10 to 100 trillion microorganisms in the human gut, called the gut microbiota, which combined with their genetic material, making up the gut microbiome [25]. The bacteria in the gut microbiota are dominated by *Gram-positive Firmicutes* and *Gram-negative Bacteroidetes* [26]. The gut microbiome maintains gut homeostasis by assisting in nutrient digestion, metabolism, immune function, and barrier protection and is therefore considered a functional organ. The exact function of the gut microbiota remains largely unknown. However, it plays an important role in the processing of complex indigestible polysaccharides from short-chain fatty acids, providing energy for the host, and also participating in the synthesis of vitamins, bile acids, and amino acids; the metabolism of drugs and toxins; and the integrity of the intestinal barrier. Although the gut microbiome is already formed at age 3 years, a variety of factors that may alter its diversity over the course of a person's life, including medications, geography, stress, and diet. Using 16S rRNA sequence analysis, differences in bacterial community structure were found in humans eating different diets [27]. Specifically, the term “dysbiosis” refers to any imbalance between beneficial and pathogenic bacteria or alterations in the taxonomic composition and function of the gut microbiota. In both mice and humans, the abundance of *Firmicutes* and *Bacteroidetes* varies with body fat composition, with an increase in *Firmicutes* and a decrease in *Bacteroidetes* when body fat content increases [28]. The study showed that germ-free mice, while consuming more food than conventional mice, had leaner physical characteristics and increased fat due to increased dietary energy intake after transferring fecal material from conventional mice. When humans are obese, dietary modification to restrict fat or carbohydrates shifts the gut microbiota from an “obese” to a “thin” phenotype [29]. The quantitative changes in gut microbial composition may independently associated with the development of NAFLD that caused progression to NASH and HCC. Therefore, species-specific biomes may reflect the staging of NAFLD. Although liver biopsy is still the gold standard for disease diagnosis, gut microbiota sequencing has become a noninvasive auxiliary test for NAFLD diagnosis. As a biomarker of disease phenotype or to provide prognostic value for the possible development of cirrhotic liver cancer, supplementation of probiotics to modulate the structure of the microbiota has become a potential therapeutic option for the treatment of NAFLD [30].

The article "Effect of Probiotics Therapy on Nonalcoholic Fatty Liver Disease" was published in 2022. Journal: Comput Math Methods Med.

Abnormal ALT, AST, and GGT indicators are usually used as markers of liver damage, but only as general markers of liver damage, not markers of specific liver function. In NAFLD patients, intestinal inflammation is thought to promote the translocation of bacteria and their products, which in turn stimulate Kupffer cells and stellate cells of the liver, promoting hepatic inflammation [31], leading to hepatocyte death and concomitant hepatic enzyme release, so elevated liver enzymes are considered a reliable indicator of liver damage. In the present study, the improvement of liver function in NAFLD patients after probiotics treatment was a basic marker for evaluating the therapeutic effect by quantifying clinical liver function. In addition, the level of ALT, AST, and GGT in the probiotics group was significantly lower than that in the control group, with statistical significance.

Intrahepatic lipid accumulation exhibits the effect of increased lipolysis, hepatic free fatty acid and relatively low-density lipoprotein synthesis, decreased free fat acid oxidation, and triglyceride transport, leading to lipid accumulation in the liver [32]. Intrahepatic lipid accumulation interferes with hepatic sinusoidal microcirculation and the ability of hepatocytes to clear microbial and gut-derived danger signals, enhancing the reactivity of Kupffer cells, which are critical for the progression of NAFLD [33]. In the present study, the levels of LDL-C, HDL-C, and TG in the probiotics group were significantly lower than that in the control group. Therefore, using probiotics could improve NAFLD by improving lipid status and correcting lipid metabolism.

IR is also part of a preemptive mechanism in the pathogenesis of “two-hit” nonalcoholic fatty liver disease. The effectiveness of IR in the pathogenesis of NAFLD occurs through the following mechanisms: increased activation of sterol regulatory element binding and carbohydrate response element binding protein [34]. It was revealed that probiotics supplementation is helpful to improve IR and reduce insulin levels in patients with NAFLD in the present study. In addition, the level of GLU was significantly increased in the probiotics group which indicating that probiotics may help to increase the level of GLU.

The high prevalence of NAFLD in obese people shows that obesity is one of the most important factors related to the disease, and obesity plays an important role in the development of the disease to NASH. It has shown that specific microbial species are related to the reduction or increase of body weight. Previous studies demonstrated that surgical resection of intra-abdominal fat can reverse liver IR and steatosis while [35]. Therefore, the clinical evaluation of BMI improvement after probiotics treatment is a useful index of treatment effect among NAFLD patients. During the progression of NAFLD, inflammation through the activation of nuclear factor kappa-B (NF-*κ*B) and mitogen-activated protein kinase (MAPK) pathways increases the activity of Kupffer cells and aggravates the progression of liver and systemic inflammation. Studies have shown that the severity of NAFLD is directly related to the levels of inflammatory markers such as TNF-*α* and CRP [36]. Elevated levels of free fatty acids in the liver provide a source of oxidative stress, which is an important cause of the development of steatosis to steatohepatitis. TNF-*α* is a pleiotropic cytokine that activates multiple signaling mechanisms leading to hepatocyte apoptosis, hepatic stellate cell activation, and hepatic cell aggregation [37]. In the present study, it was showed that the levels of BMI, TNF-*α*, and CRP are significantly induced in the probiotics group. The possible reason is that intrahepatic free fatty acids have direct cytotoxic effects, increasing lysosomal permeability and hepatocyte synthesis of TNF-*α* [38]. However, according to the probiotics therapy, the levels of free fatty acids were inhibited which leads to positive effect on NAFLD.

The article "Effect of Probiotics Therapy on Nonalcoholic Fatty Liver Disease" was published in 2022. Journal: Comput Math Methods Med.

Although the molecular mechanism of probiotics has not been fully elucidated, current studies suggest that probiotics in the treatment of NAFLD may modulating the composition of intestinal flora, improving the permeability of intestinal mucosa, inhibiting the inflammatory response, and regulating the immune system by probiotics. It was found that several strains of *Bifidobacterium* may produce bacteriocin-like compounds that are toxic to both Gram-positive and Gram-negative bacteria. Furthermore, some secreted probiotic factors are able to inhibit the binding of pathogenic bacteria to specific receptors expressed on the epithelial surface except the antibacterial effects [39]. Several strains of *Lactobacillus* and *Bifidobacterium* are able to compete with and displace pathogenic bacteria including *Staphylococcus aureus*, *Clostridium difficile*, *Enterobacter aerogenes*, *Listeria Special bacteria*, and *Salmonella enterica* [40]. Therefore, probiotics may improve the intestinal ecology and microbial composition to compete and replace with pathogenic bacteria and prevent the overgrowth of small intestinal bacteria. As the incidence of NAFLD continues to rise, research into therapeutic approaches to mitigate the occurrence and progression of NAFLD remains essential [41]. More and more researches are expanding our understanding of the mechanisms by which NAFLD is affected by gut microbes especially beneficial bacteria [42]. However, further well-designed prospective clinical studies combined with preclinical models are needed to establish pathogenic microbe-host interactions in the pathogenesis of NAFLD. Therefore, we hope that the intestinal microbiome will become an indispensable part of personalized medicine, especially in multifactorial chronic metabolic diseases such as NAFLD in the next few years. Previous research shows that dietary and lifestyle changes have been shown to improve NAFLD disease markers, but patient compliance has been problematic, making treatment limited [43]. With increasing research on the gut microbiota and its role in obesity and liver disease, fecal microbial signatures can serve as noninvasive diagnostic tools or provide prognostic value [44], and future research directions are to use the gut microbiota as a treatment options for NAFLD.

The article "Effect of Probiotics Therapy on Nonalcoholic Fatty Liver Disease" was published in 2022. Journal: Comput Math Methods Med.

## 5. Conclusion

Gut dysbiosis is a risk factor that may influence and contribute to the pathogenesis of NAFLD. The ability of probiotics to reverse gut dysbiosis has generated increasing interest in investigating probiotics as an alternative treatment option for patients with NAFLD. In the present study, it was found that probiotics supplementation has a significant positive effect on the treatment of NAFLD. In addition, probiotics supplementation plays a positive role in improving patients' lipid metabolism, reducing IR, regulating body immunity, improving liver function, and delaying disease progression in the treatment of NAFLD. In this growing area of NAFLD-related therapeutic research, further research is needed to more clearly elucidate the role of probiotics.

## 6. Limitations of the Study

(1) All the included literatures and studies were randomized controlled trials, but some trials did not accurately explain the random sampling method, distribution scheme, and blind method. (2) The gold standard for the diagnosis of NAFLD is normal liver biopsy, but few studies are based on ultrasound, MRI, and biochemical indexes. (3) A few of included articles have obvious heterogeneity, which may be related to the information bias in the process of data collection, the area of the included population, the type, the dose, the treatment time, and the duration of the disease. Therefore, the therapeutic effect of probiotics in the treatment of NAFLD still needs to be confirmed by further randomized double-blind controlled trials. (4) The actual action mechanism of probiotics in NAFLD and the efficacy of NAFLD in children and adults are different. (5) The comparison of the efficacy of effective probiotics, the specific action targets of each probiotic, and the long-term efficacy have not been elucidated well.

## Figures and Tables

**Figure 1:** Flow chart of the study selection process.

**Figure 2:** Forest plots of the effect of probiotics therapy on (a) ALT, (b) AST, and (c) GGT levels.

**Figure 3:** Forest plots of the effect of probiotics therapy on (a) TG, (b) LDL-C, and (c) HDL-C levels.

**Figure 4:** Forest plots of the effect of probiotics therapy on (a) IR, (b) insulin, and (c) GLU levels.

**Figure 5:** Forest plots of the effect of probiotics therapy on (a) BMI, (b) TNF, and (c) CRP levels.

**Figure 6:** Funnel plots for publication bias analysis of the included articles.

The article "Effect of Probiotics Therapy on Nonalcoholic Fatty Liver Disease" was published in 2022. Journal: Comput Math Methods Med.

**Table 1:** Basic traits and characteristics of the included studies.

First author	Country	Publication years	Case number	Intervention time	Diagnostic method	Probiotic ingredients	Control group	NOS
Abdel [45]	Egypt	2017	30 (15/15)	4 weeks	Liver biopsy	Lactobacillus	Nonplacebo	5
Abhari [46]	Egypt	2020	45 (23/22)	12 weeks	N/A	Bacillus	Placebo	6
Ahn [47]	South Korea	2019	65 (30/35)	12 weeks	Liver biopsy	6 probiotic mixtures	Placebo	7
Alisi [48]	Italy	2014	24 (10/14)	4 months	Liver biopsy	VSL #3	Placebo	8
Aller [49]	Spain	2011	28 (14/14)	3 months	Liver biopsy	Lactobacillus bulgaricus, Streptococcus thermophilus	Placebo	6
Asgharian [50]	Iran	2016	74 (36/38)	12 weeks	Ultrasonic examination	Lactobacillus, Bifidobacterium, Streptococcus	Placebo	8
Bakhshimoghaddam [51]	Iran	2018	68 (34/34)	24 weeks	Ultrasonic examination	Streptococcus thermophilus, Lactobacillus, Bifidobacterium	Nonplacebo	9
Behrouz [52]	Iran	2017	60 (30/30)	12 weeks	Ultrasonic examination	Lactobacillus, Bifidobacterium	Placebo	7
Cai [53]	China	2020	140 (70/70)	12 weeks	Liver biopsy	Lactobacillus, Bifidobacterium, Enterococcus	Nonplacebo	6
Dagan [54]	Israel	2017	80 (40/40)	24 weeks	N/A	Lactobacillus, Bifidobacterium, Streptococcus, Lactococcus	Placebo	6
Duseja [55]	India	2019	30 (17/13)	48 weeks	Liver biopsy	Lactobacillus, Bifidobacterium	Placebo	5
Ekhlasi [56]	Iran	2016	30 (15/15)	8 weeks	Ultrasonic examination	Lactobacillus, Bifidobacterium, Streptococcus	Placebo	6
Eslamparast [57]	Iran	2014	52 (26/26)	28 weeks	Ultrasonic examination	Lactobacillus, Bifidobacterium, Streptococcus	Placebo	7
Ferolla [58]	Brazil	2016	50 (27/23)	12 weeks	Liver biopsy	Lactobacillus	Nonplacebo	7
Famouri [59]	Iran	2017	64 (32/32)	12 weeks	Ultrasonic examination	Lactobacillus, Bifidobacterium	Placebo	7
Javadi [60]	Iran	2017	38 (19/19)	18 weeks	Liver biopsy	Bifidobacterium longum, Lactobacillus acidophilus	Placebo	6
Kobyliak [61]	Ukraine	2018	58 (30/28)	8 weeks	Liver biopsy	Bifidobacterium, Lactobacillus, Lactococcus, Propionibacterium	Placebo	7
Malaguarnera [62]	Italy	2012	66 (34/32)	24 weeks	N/A	Bifidobacterium longum	Placebo	6
Manzhalii [63]	Germany	2017	75 (38/37)	12 weeks	Ultrasonic examination	Lactobacillus casei, L. rhamnosus, L. bulgaricus, Bifidobacterium longum, and Streptococcus thermophilus	Nonplacebo	7
Mofidi [64]	Iran	2017	42 (21/21)	28 weeks	Ultrasonic examination	Lactobacillus, Bifidobacterium, Streptococcus	Placebo	6
Nabavi [65]	Iran	2014	72 (36/36)	18 weeks	Ultrasonic examination	Lactobacillus bulgaricus and Streptococcus thermophilus	Placebo	6
Sepideh [66]	Iran	2015	42 (21/21)	8 weeks	Ultrasonic examination	Lactobacillus, Bifidobacterium, Streptococcus	Placebo	5
Shavakhi [67]	Iran	2013	63 (32/31)	6 months	Liver biopsy	Protexin tablet	Placebo	5
Vajro [68]	Italy	2011	20 (10/10)	8 weeks	Ultrasonic examination	Lactobacillus	Placebo	6

The NOS presents Newcastle-Ottawa Scale.

The article "Effect of Probiotics Therapy on Nonalcoholic Fatty Liver Disease" was published in 2022. Journal: Comput Math Methods Med.

**Table 2:** Related factors for probiotics therapy on NAFLD patients.

Related factors	MD	95% CI	*P* value
ALT	-7.25	-10.11–-4.39	0.00001
AST	-3.53	-5.62–-1.44	0.0009
GGT	-2.27	-4.49–-0.05	0.04
TG	-0.42	-0.53–0.05	0.01
LDL-C	-1.38	-2.15–-0.60	0.0005
HDL-C	-19.92	-30.56–-9.29	0.0002
IR	-0.61	-1.02–-0.21	0.003
Insulin	-1.27	-2.39–-0.15	0.03
GLU	-0.03	-0.32–0.25	0.82
BMI	-0.80	-1.51–-0.08	0.03
TNF-*α*	-2.43	-6.56–1.71	0.03
CRP	-1.06	-1.94–0.18	0.02

## Data Availability

All data included in this study are available upon request by contact with the corresponding author.

## Abbreviations

ALT: Alanine aminotransferase
AST: Aspartate aminotransferase
BMI: Body mass index
GLU: Blood glucose
CRP: C-reactive protein
IR: Insulin resistance
LDL-C: Low density lipoprotein
MAFLD: Metabolic fatty liver disease
GGT: *γ*-Glutamyltransferase
NASH: Nonalcoholic steatohepatitis
NAFL: Nonalcoholic fatty liver
NAFLD: Nonalcoholic fatty liver disease
TNF-*α*: Tumor necrosis factor-*α*
TG: Triglyceride.
